This article has been retracted.

# Simulation Analysis and Control of Multi-energy System for Fuel Cell Hybrid Electric Vehicle Based on Wavelet Transform

**DOI:** 10.1155/2022/3011307

**Published:** 2022-07-14

**Authors:** Mengjie Li, Qianchao Liang, Jinyi Hu, Yifan Liang, Jianfeng Zhao

**Affiliations:** Department of Power Engineering, Naval University of Engineering, Wuhan, Hubei 430033, China

## Abstract

In order to address the issue of multi-energy system fuel cells having a short life cycle and low fuel efficiency, a Fuel Cell Hybrid Vehicle was developed. The goal of this research is to use wavelet transformation to simulate, evaluate, and regulate the multi-energy system of a fuel cell hybrid car. To begin, a hybrid model of the fuel cell and an overall dynamic model of the fuel cell, as well as a DC/DC converter model, are constructed in accordance with the simulation environment. Second, the hybrid vehicle system's power information is successfully captured, and the power signal acquired is processed using the wavelet transform. The fuel cell power control and the composite power supply's power allocation module are independently input into the hybrid system's low frequency and high frequency power requirements. PI control is used to regulate the power of the storage device in the hybrid power system, as well as the power settings of the output fuel cell and supercapacitor. The simulation results show that the power battery fluctuation range of the hybrid vehicle multi-energy system based on the wavelet transform proposed in this paper is significantly smaller than that of other methods, and the entire process operates at low power points. The results of the experiments suggest that the strategies given in this study can successfully extend the life of fuel cells while also lowering the overall fuel efficiency of the vehicle system.

## 1. Introduction

Wavelet transform is assumed to be an effective approach which has the capability to divide, separate a single & powerful signal into a group of multiple signals probably with lower power as compared to the original. However, during that transformation it tries to retain up to maximum possible level that the controlling of two measures, i.e., shifting & scaling respectively, particularly of the powerful single source signal. Or simply it can be perceived as a mathematical model for the transformation of single power signal into multiple signal to improve its functionality and usability of the resources. Apart from it, this approach has the built in capacity to extract in an effective manner both the temporal and spectral transformation, specifically local in this case, that is also assume to be its realist and major breakthrough than other transformation techniques which are available.

Environmental pollution and energy crisis have become the focus of global attention and have a direct impact on the national ecological sustainable development. Therefore, all countries around the world attach great importance to environmental and energy issues. Automobiles cause environmental pollution and high energy consumption. Researchers in the automotive industry must seek for renewable and new energy sources, and take a series of measures to improve the economy of automotive fuel, such as new technologies, new materials and new processes, in order to reduce automotive exhaust emissions. In recent years, every country is developing green automobile technology with high efficiency and low pollution. Well-known automotive companies have improved the internal combustion engine technology of traditional fuels, and on the basis of improving the fuel combustion efficiency, using different catalysts to reduce harmful components after fuel combustion, effectively reducing the ecological environment pollution. However, internal combustion engine automobiles can not effectively solve these problems, so the automotive industry has carried out in-depth research on new environmentally friendly automobiles.

The growth of electric cars will aid in the diversification of transportation energy structures, the reduction of petroleum resource scarcity and the bad impact of fuel automobile emission pollution, and the promotion of China's automotive industry's leap-forward development. An electric car may be considered a green mode of transportation. The qualities of a battery hybrid car, which primarily employs hydrogen power generation as a power source, include zero emissions, high energy conversion efficiency, and low noise. Hydrogen is a type of secondary energy that may be derived from a variety of sources. The present automobile industry is focusing on the development of fuel cell hybrid vehicles. The multi-energy system analysis and control of a fuel cell hybrid electric vehicle are thoroughly investigated in this work.

The following are the paper's innovations: (1) A hybrid fuel cell model, a dynamic model, and a DC/DC converter model are developed using the simulation environment, and the wavelet transform is used to assess and operate the multi-energy system of a fuel cell hybrid electric vehicle. (2) When compared to previous ways, the methods proposed in this research can successfully extend the life of fuel cells while lowering the overall fuel efficiency of the vehicle.

The remaining parts of the article are given as below.

A survey of those technique which are assumed to be linked to the problem under consideration is reported in section 2 of the paper. In this, we have worked on how these systems are able to solve a problem and why these are not applicable to resolve this problem, i.e., which is considered in this paper. Section three of the paper is dedicated to the fuel cell hybrid electric vehicle system model where we have described how these vehicle could be make more efficient and their fuel adjustment and utilization plan could be improved extensively. Analysis and control of multi-energy system for fuel cell hybrid electric vehicle based on wavelet transform along with detailed description is presented in section four of the article. Results and discussion are provided in subsequent section where summary is given at the end.

## 2. Related Work

Famous automotive manufacturers from across the world are working on a variety of electric vehicles and have achieved significant progress and achievements. W. Li et al. A hybrid vehicle energy management system based on deep reinforcement learning is presented to increase fuel efficiency and battery life cycle of fuel cell hybrid automobiles. This approach initially adds a life factor to the reward signal to lessen the fuel cell's power fluctuation, which can extend the battery's life cycle. Using the limited motion space approach, the fuel cell's power system operates within a high-efficiency range, boosting the overall efficiency of the automotive power system and allowing for offline training under various operating situations. Experiments reveal that when compared to standard techniques without a life factor, this method has a quicker convergence speed, greater stability, and can effectively lower the power consumption of fuel cells, which can assist to extend the life of fuel cells. Despite the fact that the life of fuel cells extends under variable operating circumstances, the overall fuel efficiency is poor [1]. A hierarchical energy control system for fuel cell and supercapacitor energy allocation in fuel cell hybrid cars is presented by Li Z H et al. The method is divided into two layers: the upper part uses the fuel cell and SOC value to design a rule control strategy to continuously optimise the fuel cell's energy output, and the lower part uses the battery supercapacitor's characteristics to design a sliding filter to keep the battery's energy output stable. Experiments are conducted in a virtual setting. When compared to standard ways, the experimental findings suggest that this strategy may effectively improve fuel cell efficiency by distributing energy output sensibly. However, this approach has the disadvantage of a shorter fuel cell life cycle [2]. Cui P F et al. propose a fuzzy control-based energy control technique for fuel cell hybrid power systems. The fuel cell can run within the limited power supply range thanks to the fuzzy controller's membership function and fuzzy rule design. The cumulative power increment of the fuel cell is used to continually optimise the fuel cell's power, and the hybrid power system is chosen based on the fuel cell hybrid power system's selection. The simulated hybrid power system model is created and compared with the finite state method under cyclic conditions in a simulated experimental scenario. The findings of the research suggest that this approach can secure the fuel cell's life cycle through power distribution, but it has an issue with low fuel efficiency [3]. Tan Y et al. provide a hybrid technique for energy control of fuel cell hybrid power systems based on supercapacitor and fuzzy control. An enhanced energy control strategy is presented using regular batteries as auxiliary batteries. Supercapacitors offer a high power density and energy density, allowing them to handle the power demands of hybrid cars more effectively. The conventional power control technique has been scientifically updated, and the hybrid power system is controlled by a fuzzy control approach, which enhances fuel economy by satisfying the power vehicle system's power performance. This approach, however, has the drawback of a shorter fuel cell life cycle [4].

## 3. Fuel Cell Hybrid Electric Vehicle System Model

The hybrid vehicle system model of fuel vehicle is roughly divided into three modules, namely, energy management system, hybrid power system and vehicle dynamics model. On the basis of describing the hybrid power system of the fuel cell vehicle, a fuel cell vehicle model [5, 6] is built using the simulation platform. The basic parameters of fuel cell automobiles are shown in Table 1.

### 3.1. Power System of Fuel Cell Hybrid Vehicle

A hybrid vehicle multi-energy system with fuel cells employs a fuel cell and power battery hybrid powertrain system.  Figure 1 depicts the system's general structural principle. Fuel cell modules and power batteries, as well as DV/DC branch converter modules, may be shown in Figure 1. The fuel cell is the primary power source, the accumulator is the auxiliary power supply, and the DC/DC converter is the voltage output that the fuel cell voltage is steady within the bus voltage value [7, 8].

### 3.2. Fuel Cell Model

Currently, the common fuel cell models are generally divided into three types: chemical model, experimental model and electrical model. The electrical model simplifies the fuel cell by using equivalent circuit to simulate the performance of the fuel cell, but does not consider other aspects. In this paper, the equivalent circuit model is used to scientifically simulate the fuel cell [9, 10].

The equivalent model of a fuel cell can be expressed as:

(1) $$\begin{array}{c} E_{fc}=E_{oc}-N\cdot A\cdot 1n\left(\frac{i_{fc}}{i_{o}}\right)\cdot i_{fc}\cdot r_{f\text{cin}}. \end{array}$$

Formula (1), *N* denotes the number of fuel cells, *r*_*fcin*_ denotes the resistance of the fuel cells, and the output voltage of the fuel cells is mainly determined by the input current *i*_*fc*_ and some parameters such as open circuit voltage *E*_*oc*_, Tafir slope *A* and exchange current *i*_*o*_.

### 3.3. Power Battery Model

The power battery model and the fuel cell model are the same, they contain many models. This paper mainly takes the equivalent circuit model, considers the accuracy and the hardware conditions of the computer, and selects *R*_int_.

The mathematical model of the power battery is expressed as:

(2) $$\begin{array}{c} E_{\text{bat}}=n\cdot \left(E_{m}-I_{\text{bat}}\cdot R_{\text{bat}}\right). \end{array}$$

In formula (2), *E*_bat_ denotes battery end voltage, *E*_*m*_ denotes battery open-circuit voltage, *I*_bat_ denotes battery current, *R*_bat_ denotes battery resistance, *n* denotes number of power batteries as a single unit.

The power battery SOC calculation is expressed as:

(3) $$\begin{array}{c} SOC\left(t\right)=SOC\left(t_{0}\right)+\frac{I_{\text{bat}}\cdot \Delta t}{C_{\text{bat}}}. \end{array}$$

In formula (3), *SOC*(*t*) represents the current power battery capacity, *SOC*(*t*_0_) represents the initial battery capacity, and *C*_bat_ represents the rated capacity.

### 3.4. DC/DC Converter Model

The principle of DC/DC converter is shown in Fig.  2. In Figure 2, the output voltage of the fuel cell will change greatly during operation, and the DC / DC converter must be used to reduce voltage and stabilize voltage. The DC / DC DC converter in the DC / DC DC converter model is buck type, using the actual measured *i*_*fc*_ and the reference output current *i*_*fc*_−_*ref*_ difference regulates the duty cycle of DC / DC converter, so as to reduce the fuel cell voltage into DC bus voltage [11, 12].

## 4. Analysis and Control of Multi-Energy System for Fuel Cell Hybrid Electric Vehicle Based on Wavelet Transform

Energy system analysis and control mainly consists of three parts, which are the control of wavelet transform, energy storage equipment and power protection strategies. The control structure diagram based on the wavelet transform is shown in Figure 3. In Figure 3, *S*_bat_ represents the charge state of the fuel cell, *S*_bat_−_ref_ represents the set value of the charge state of the fuel cell, *V*_*sc*_ represents the voltage of the supercapacitor, *V*_*sc*_−_*ref*_ represents the set voltage of the supercapacitor, *P*_bat_−_ref_ represents the set value of the battery output power, *P*_*fc*_−_*ref*_ represents the set value of the output power of a fuel cell, *P*_*sc*_−_*ref*_ represents the output power setting of the supercapacitor [13, 14].

### 4.1. Sliding Window

Today, the effective functionality of the automatic system is assumed to effective and could be more increase if the well-known concept of the sliding windows is utilized in it. This approach is based on the idea of changing or constantly updating the matching or active window based on the requirement of the problem and system which is needed to be developed. Additionally, size of the sliding window is very crucial as it is not only a way forcing the system to work on the most recent set of data values but it is also vital for effective decision making process.

A sliding window is used to complete the control of the hybrid vehicle system based on the wavelet transform. Sliding window is mainly based on brake unit length enclosing time series, comprehensive calculation of enclosing time series, reasonable sliding with fixed length slider, sliding a unit, can feedback the information contained in it [15, 16].

Set the time window to set the amount of data is 2^*p*^ (*p* must be a positive integer), and set the time *i* collection fuel cell hybrid vehicle energy data series is *a*_1_, *a*_2_,…, *a*_*i*_, the actual steps of filtering using sliding window method are as follows.

1. When *i*≺2, because the amount of data sampled from the hybrid vehicle is less than that required by the sliding window, the wavelet transform operation cannot be carried out, and the output value is the current sampling value *a*_*i*__._
2. When *i*=2^*p*^, the data amount needed to reach the sliding window is sampled for hybrid vehicles. The first wavelet transformation is carried out. The original fuel cell power system data series are *a*_1_, *a*_2_,…, *a*_*i*_. After transformation, the data series can be recorded as *a*_1_^*∗*^, *a*_2_^*∗*^,…, *a*_*i*_^*∗*^. Since a filter transformation is performed, *a*_*i*_^*∗*^ is used as the output value for the current moment [17, 18].
3. When *i*=2^*p*^+1, the sliding time window can shift one position to the right, and carry out the wavelet transformation on *a*_2_, *a*_3_ …, *a*_2^*p*^+1_. After the transformation, the data sequence is *a*_2_^*∗*^, *a*_3_^*∗*^,…, *a*_2^*p*^+1_^*∗*^, *a*_2^*p*^+1_^*∗*^ as the output value of the current moment.
4. Repeat these three steps

The fuel cell related data in the sliding window is updated continuously with the information collected by the sensor, and then the related data in the window is transformed by wavelet transform, and the value transformed is treated as the output of the wavelet transform. After several simulation debugging, the time scale size is selected as 16.

### 4.2. Wavelet Transform

Wavelet transform, as described above, is an effective way of dividing a single, preferably large, signal into multiple low level signal while preserving scaling factors along with other. As it is a mathematical model where solid justification is available and is proved by researcher individuals and developers. The information of the sliding window is extracted effectively by using the wavelet transform and decomposed according to different phases and scales. The power requirement of multi-energy system of hybrid electric vehicle is treated as discrete signal. The discrete power requirement signal is decomposed into different decomposition layers by discrete wavelet decomposition function and reconstruction function. The formulas of discrete wavelet transformation and inverse transformation for fuel cell hybrid vehicle are expressed as follows:

(4) $$\begin{array}{c} W\left(\lambda ,r\right)=\int x\left(t\right)\frac{1}{\sqrt{\lambda }}\psi \left(\frac{t-r}{\lambda }\right)\text{d}t, \end{array}$$

(5) $$\begin{array}{c} x\left(t\right)=\sum_{j\in Z}\sum_{k\in Z}W\left(j,k\right)\psi_{j,k}\left(t\right). \end{array}$$

In formulae (4), (5), *λ* Represents the scale factor of the hybrid power system. *λ*=2^*j*^, *r* denotes the shift factor of the hybrid system, *r*=*k*2^*j*^, *x*(*t*) denotes the original signal, *ψ* representation parent function.

Compared with other common wavelets, the Haar wavelet mother function has the same advantages in time domain as the shortest filter span and the wavelet transform and inverse transform, because these characteristics make the Haar wavelet transform easier to control in hybrid power systems. The Haar wavelet transform expression is expressed by formula (6) when the simplified program improves the program execution efficiency:

(6) $$\begin{array}{c} \psi \left(t\right)=\left\{\begin{array}{c} \begin{array}{cc} 1 & t\in \left[0,1/2\right], \end{array}\\ \begin{array}{cc} -1 & t\in \left[1/2,1\right]\text{else,} \end{array}\\ \begin{array}{cc} 0 & \text{else}. \end{array} \end{array}\right. \end{array}$$

Using *N*-channel wavelet transformation, the original information signal *x*(*t*) is decomposed into reference signal and detail signal by low-pass and high-pass filtering, and reconstructed by reconstruction filter.

Since the fuel cell is an outward power output, it cannot absorb the energy. According to formula (7), the positive power of the low frequency signal is assumed, while the power of the composite power supply is assumed, while the decomposed high frequency power demand is assumed by the composite power supply.

(7) $$\begin{array}{c} P_{fc_{-}ref}=\left[\begin{array}{c} \begin{array}{cc} x_{0}\left(n\right), & x_{0}\left(n\right)≻0, \end{array}\\ \begin{array}{cc} 0, & \text{else}. \end{array} \end{array}\right] \end{array}$$

### 4.3. Power Distribution for Composite Power Supply

According to the composite power control method, the control method is composed of support vector machine and low-pass linear filter. Composite power supply can be divided into low frequency and high frequency by filter, high frequency by supercapacitor, low frequency by lithium battery. Hybrid vehicle can select No. 1 low-pass filter at stable speed, Hybrid vehicle can select No. 2 low-pass filter at dynamic condition, and select low-pass filter at steady speed and in dynamic condition can be expressed as:

(8) $$\begin{array}{c} L_{d}\left(s\right)=\frac{1}{T_{1}s+1}, \end{array}$$

(9) $$\begin{array}{c} L_{j}\left(s\right)=\frac{1}{T_{2}s+1}. \end{array}$$

In formulas (8), (9), *T*_1_, *T*_2_ the time constant representing the filter. The power allocation of a fuel cell hybrid vehicle system can be controlled by the time constant *T* of the adjustment filter. The higher the time constant value, the lower the power requirement of the high frequency using the low-pass filter [19, 20].

### 4.4. Power Control of Energy Storage Devices

The power status of batteries and supercapacitors in the composite power supply of fuel cell hybrid vehicle multi-energy system can be controlled by PI control method. As shown in Figure 4, the power control input of lithium batteries is the difference between batteries setting SOC and batteries monitoring SOC, and the charging power of output power batteries is *P*_charge_−_bat_.

When controlling the electric quantity of super capacitor, the super capacitor voltage control method is better than the super capacitor SOC control method. As shown in Figure 5, the super capacitor control input of the fuel cell hybrid electric vehicle system is the difference between the capacitor voltage and the detection capacitor voltage, and the charging power of the output capacitor is *P*_charge_−_sc__._

When the power demand of the fuel cell hybrid electric vehicle system fluctuates greatly, the influence of power control on the power distribution control of the filter can be ignored. When the power demand of the fuel cell hybrid electric vehicle system is very small, this control method can realize the scientific control of the power of super capacitor and lithium battery, so that the power of battery and super capacitor can be maintained within a reasonable range.

### 4.5. Protection of Energy Storage Equipment

If the power battery in a fuel cell hybrid electric vehicle system discharges electricity at a low power level, the battery's service life will be harmed. Battery damage and even spontaneous combustion might occur if the battery is still charging at high power. The operation of the DC / DC voltage converter will be affected if the super capacitor in the composite power supply releases power when the power is low, compromising the overall stability of the fuel cell hybrid vehicle system. When the power is strong and the super capacitor is still charging, it is simple to trigger an explosion, which is extremely dangerous. As a result, when implementing a hybrid power supply system in practise, a hybrid power supply protection plan must be developed.

The power of super capacitor and battery charging is provided by fuel cell, and the output power of fuel cell is expressed as:

(10) $$\begin{array}{c} P_{fc}=\min\left[P_{\text{load}}+P_{{\text{charge}}_{-}\text{bat}}+P_{{\text{charge}}_{-}\text{sc}},P_{fc\;\max}\right]. \end{array}$$

Through the above process, the multi energy system analysis and control of fuel cell hybrid electric vehicle based on wavelet transform are completed.

## 5. Analysis of Experimental Results

The multi energy system simulation experiment of fuel cell hybrid electric vehicle is carried out by using MATLAB simulation platform. An economic car with independent property rights is selected as the simulation model, which is a precursor model.  Table 2 shows the specific parameters of the simulation model.

According to the hybrid electric vehicle system control method based on wavelet transform proposed in this paper and the hybrid electric vehicle system control method based on deep reinforcement learning proposed in literature [1], the SOC curve of power battery is simulated and shown in Figure 6.

Through the analysis of Figure 6, it can be seen that the two hybrid system controls can ensure that the power battery SOC is maintained at a normal level, but the whole process fluctuation range of power battery SOC based on wavelet transform is relatively smaller than that based on deep reinforcement learning control method. At the same time, the difference between the initial value and the final value of SoC Based on wavelet transform is less than that based on deep reinforcement learning control method, which is compared with that based on deep reinforcement learning control method. The method proposed in this paper can effectively prolong the battery life and reduce the number of battery replacement, so as to reduce the economic cost of multi energy system of hybrid electric vehicle.

The output power curve *P*_*fc*_ of fuel cell obtained from the hybrid electric vehicle system control method based on wavelet transform and the hybrid electric vehicle system control method based on deep reinforcement learning proposed in reference [1] is shown in Fig.  7. In order to analyze the simulation results shown in Figure 7, according to the factors affecting the life of fuel cell, four indexes in Table 3 are extracted to measure the impact of hybrid electric vehicle multi energy system on the life of fuel cell under two different control methods.

Through the analysis of Figure 7 and Table 3, it can be seen that under the control of hybrid electric vehicle system based on deep reinforcement learning, the fuel cell works at the low power point for half of the overall working time, while under the control of hybrid electric vehicle system based on wavelet transform, the fuel cell works at the low power point throughout the whole process. In addition, compared with the control method based on deep reinforcement learning, Compared with the method of enhancing the working cycle of the hybrid power system in this paper, the working time of the proposed method can be significantly prolonged.

In the multi energy system of hybrid electric vehicle based on wavelet transform, the bus current, the output current of fuel cell and the output current of power cell are shown in Figure 8.

Through the analysis of figure 8, it can be seen that the multi-energy system of hybrid electric vehicle based on wavelet transform can control the flow of energy between fuel cell and power cell and load, and the hybrid power source of fuel cell and power cell can meet the power demand of load, so as to ensure the stable operation of multi-energy system of hybrid electric vehicle.

## 6. Conclusion

The theory of wavelet transform is applied to the multi energy system of fuel cell hybrid electric vehicle, and the structure design and simulation analysis of hybrid electric vehicle system are carried out. Additionally, sliding window based concept is utilized to make the system more effective and to focus on the most recent data values which are vital for the effectiveness of a systems. The simulation results show that the multi energy system of hybrid electric vehicle based on wavelet transform can not only control the energy flow of the power system, but also prolong the service life of fuel cell compared with other control methods, so as to reduce the economic cost of fuel cell hybrid electric system.

In future, the proposed system could be possibly be extended to integrate newly developed methodology along with the sliding window based concept to make these system effective and robust.

## Figures and Tables

**Figure 1:** Fuel cell hybrid power system structure.

**Figure 2:** schematic diagram of DC/DC DC converter.

**Figure 3:** Energy control strategy structure.

**Figure 4:** Battery power control policy.

**Figure 5:** Power control policy for the supercapacitor.

**Figure 6:** Comparison of SOC curves of power batteries with different methods.

**Figure 7:** Output power curves of fuel cells with different methods.

**Figure 8:** Bus current, fuel cell and power cell output current curves.

**Table 1:** Basic parameters of fuel cell vehicles

Parameter	The numerical
Automobile mass/kg	1624
Rated power of fuel cell/kW	85.5
Fuel cell open circuit voltage/V	400
Number of fuel cells/unit	400
Maximum power of fuel cell/kW	100
Power battery capacity/Ah	13.8
Maximum power of motor/kW	100
Maximum motor speed/rpm	12500

**Table 2:** Specific parameters of simulation models

Parameter	The numerical	Parameter	The numerical
Coefficient of air resistance/CD	0.3	The front axle load/kg	540
Windward area FA/m^2^	2	The wheelbase/m	2.335
Coefficient of rolling resistance	0.01	Vehicle readiness quality/kg	895
The rolling radius of the tire is R/m	0.232	The biggest quality/kg	1270
Maximum engine power/kW	48	Accessory power load/w	700

**Table 3:** Quantitative analysis indexes of influencing factors of fuel cell life.

Indicators	Decision criteria	Time/s or times	
		The wavelet transform	Deep reinforcement learning
Operate at low power points	*P*_*fc*_≺5*kw*	0	208
Operate at high power points	*P*_*fc*_≻20*kw*	18	46
High power change rate	(*dP*_*fc*_)/(*dt*)≻80*w*/*s*	25	37
Start-stop frequency	From start to stop for a start stop	0	0

## Data Availability

The data used to support the findings of this study are available from the corresponding author upon request.
